The article "A Simple Framework of Smart Geriatric Nursing considering Health Big Data and User Profile" was published in 2020. Journal: Comput Math Methods Med.

# A Simple Framework of Smart Geriatric Nursing considering Health Big Data and User Profile

**DOI:** 10.1155/2020/5013249

**Published:** 2020-10-16

**Authors:** Shijie Li, Yongchuan Tang

**Affiliations:** ^1^Department of Critical Care Medicine, The First Affiliated Hospital of Chongqing Medical University, Chongqing 400016, China; ^2^School of Big Data and Software Engineering, Chongqing University, Chongqing 401331, China

## Abstract

The National Bureau of Statistics of China shows that the population over 65 years old in China exceeds 166 million accounting for 11.93% of the total population by the end of 2018. The importance and severity of taking care of the elderly are becoming increasingly prominent. High-quality and meticulous care for the daily life of the elderly needs helpful and advanced sciences and technologies. Smart geriatric nursing is a must. Basing on the professional knowledge of geriatric nursing, this paper proposes a framework of smart geriatric nursing which consists of three aspects of smart nursing: smart geriatric nursing in physical health using biosensor and advanced devices, smart geriatric nursing in mental health based on user profile, and smart geriatric nursing for daily life based on big data in health. The deployment of the proposed method relies on the technologies of the Internet of Things (IoT), user profile system, big data, and many other advanced information technologies. The framework of methods can provide a useful reference for the systematic technical scheme of smart geriatric nursing in an aging society.

## 1. Introduction

As a national strategy of China, Healthy China (2019-2030) program is related to the health and happiness of 1.4 billion Chinese people [1]. The program clearly shows that all Chinese people must fully implement the elderly health-promoting activity. The National Bureau of Statistics of China shows that the population over 65 years old in China exceeds 166 million accounting for 11.93% of the total population by the end of 2018. The sense of caring the elderly has become an important consensus of the whole society. High-quality and meticulous care for the daily life of the elderly needs the help of intelligent technologies [2]. This paper proposes a simple framework of smart geriatric nursing which consists of three aspects of smart nursing: smart physical health care, smart mental health care, and smart daily life care for the elderly.

It has been a widely accepted consensus that some advanced information technologies can be applied in health care. Advanced technologies in treatment and nursing field [3–6] include the Internet of Things (IoT) technologies [2], biosensor technologies, big data [7], and cloud computing [8–12]. With advanced information technologies, the medical efficiency and healthy living standard of the public can be improved significantly [13, 14]. Smart geriatric nursing is a must since China has become an aging society. This paper focuses on exploring and proposing a comprehensive and systematic smart geriatric nursing programs for the elderly's physical health, mental health, and daily life by adopting some of the latest concepts and technologies.

Smart geriatric nursing is based on the IoT technologies, sensors, big data, artificial intelligence, and many other advanced technologies in information society. A systematic framework of smart nursing for the elderly consists of three aspects: smart physical health care for the elderly, smart mental health care for the elderly, and smart daily life care for the elderly. The composition of the smart geriatric nursing method subsystem is shown in Figure 1. Smart geriatric nursing consists of the following three aspects. (1) Smart geriatric nursing in physical health using IoT technology [15, 16] consists of the elderly remote monitoring scheme using biosensor, the elderly medication safety scheme using radio frequency identification (RFID) technology [17], online (offline) elderly cognitive assessment, and many other intelligent nursing schemes related to physical health. (2) Smart geriatric nursing in mental health is based on user profile system technology [18]. It consists of the elderly profile system, online (offline) elderly psychological consultation (including mental state, psychological needs, and mental state analysis), and other smart nursing methods related to mental health. Many factors affect the mental health of the elderly [19, 20]. (3) Smart geriatric nursing for daily life is based on the big health data [21]. Big health data is derived from the elder's physical health, mental health, and user profile system.

The rest of this paper is organized as follows. The materials and methods in the proposed model are summarized and introduced in Section 2. The smart geriatric nursing in physical health is proposed in Section 3. In Section 4, the framework of smart geriatric nursing in mental health based on user profile is designed.  Section 5 is the smart geriatric nursing for daily life based on big data in health. Some limitations of the current work are discussed in Section 6.  Section 7 is the conclusion of this paper.

## 2. Materials and Methods

### 2.1. Technologies and Tools

The technologies and methods for smart geriatric nursing in physical health include biosensor-based devices and tools, smart medication systems, and smart nursing methods for geriatric common and chronic disease. Tools for mental health mainly include assessment scales, cultural activities, tourism projects, recreational activities, and cognitive training projects. For the elderly's daily life, technology in smart home is helpful.

### 2.2. Assessment Scales

Some assessment scales are necessary for monitoring the mental health state of the elderly. The research recommends some scales like the Geriatric Depression Scale (GDS) [22, 23], Roy Coping and Adaptation Processing Scale (CAPS-15) [24, 25], and Eysenck Personality Questionnaire (EPQ) [26]. The reliability and validity of the three scales were tested in the community residents in previous studies [23–27]. Since the test results showed a good reliability and validity for the three scales, they could effectively reflect some aspects of the mental health status for the elderly.

### 2.3. Inclusion and Exclusion Criteria of Areas

To implement the smart geriatric nursing, some advanced technologies and infrastructures should be deployed in the area. As we have known, China is a developing country, and this may be a challenge for some areas. The included cities and areas for smart geriatric nursing should meet the following criteria. (1) The 4G network covers the selected community. Of course, 5G network is much better. (2) The designated hospitals in this area should have mature technologies and devices to get the big data of the elderly for smart geriatric nursing. (3) The health big data is available. Records in the big data include the residents' physical condition, psychological condition, cognitive function status, living condition, and family economic status. (4) There are enough professional medical staffs. Many other criteria are also needed in practical application in a specific area.

## 3. Smart Geriatric Nursing in Physical Health

The smart geriatric nursing in physical health is aimed at helping the older people keep physical health by curing the disease and repairing the damaged organs. According to smart geriatric nursing in physical health, older people can get recovery from unhealthy condition, get back to normal life, keep healthy, and improve the quality of daily life. Smart geriatric nursing for physical health should be based on IoT technologies. In detail, the smart nursing strategies include but should be not limited to the following:

1. Biosensor-based real-time monitoring and remote management of geriatric physical activities and vital signs [28–31]
2. Medication safety and management with smart technologies including RFID, sensor, electronic tag, two-dimension code, and global positioning system (GPS) [32–36]
3. Smart assessment of geriatric cognitive function with online and offline methods [37–40], e.g., estimating the influence of healthy lifestyle on episodic memory among adults who have subjective memory complaints [40]
4. Smart nursing methods for geriatric common and chronic diseases [41–43]

In this section, we construct the framework of smart geriatric nursing in physical health by demonstrating two scenarios. The first scenario is biosensor-based real-time remote monitoring and management of geriatric physical activities and vital signs. The second scenario is medication safety and management with smart technologies.

### 3.1. Remote Real-Time Monitoring for Physical Health of the Elderly

Remote monitoring based on biosensor can be a real-time technology for smart geriatric nursing in physical health. As shown in Figure 2, the physical activities and vital signs under remote and real-time monitoring include but not limited to regular measurement of blood glucose, blood pressure measurement, cardiac function monitoring and early warning, and continuous supervision of sleep state. Smart homes can be helpful for smart geriatric nursing with the help of advanced technologies. However, it may also have a negative effect on physical functioning and cause the depression in older adults with chronic conditions [44].

An example of remote real-time monitoring for physical health of the elderly is the regular monitoring of blood glucose. The geriatric diabetic patient should follow the doctor's advice of measuring blood glucose regularly personally or with the help of a nurse according to intelligent devices. The results should be uploaded to the individual electronic medical record for smart monitoring and management. The data centre of designated medical institution records each piece of health evidence for the elderly and transfers the abnormal health data to the local community health centre where the family doctor (team), nursing staff, the elderly themselves or their relatives, and other relevant parties who have the authority to obtain the health information will be responsible for the health condition of the elderly. Smart geriatric nursing measures, such as medication reminder in voice, animation demonstration for self-care guidance, and one touch button for help, will be available whenever needed to help the elderly return to normal living condition and keep physical health by curing the disease and repairing the damaged organs. Above all, an automatic, dynamic, remote, real-time, and closed-loop monitoring and reacting system of smart geriatric nursing for physical health should be constructed to protect the health of the elderly.

### 3.2. Medication Safety and Management with Smart Technologies

Medication safety and management are a critical problem for the elderly patients [45]. The elderly is more likely to suffer from chronic diseases than the younger people. Meanwhile, medication errors are a risk factor among the elderly because of memory decay and other problems related to aging. Consequently, medication safety and management with smart technologies for the elderly are a must. A smart pill container, which is based on intelligent technologies such as RFID, sensor, wireless communication, and location, can contribute to medication safety for the elderly in cooperation with remote medication guidance whenever and wherever needed.

Smart medication systems are helpful for improving the level of geriatric nursing [46]. Firstly, it can detect drug errors quickly and easily in comparison with manual medication distribution. Secondly, it can improve safety and efficacy by ensuring that older people receive the right dose at the right time. Finally, it can reduce the burden of nursing work no matter in the hospital or at home. As shown in Figure 3, with the help of the IoT technology, especially for the sensor-related technologies, the smart pill container has the functions of flash reminding, drug dose monitoring, voice prompts, preprogrammed medication reminder, and so on. The application (APP) in a smart mobile phone is helpful for realizing the aforementioned smart geriatric nursing measure. More details on smart medicine container can be found in [47–50]. In addition, with the help of intelligent devices such as the smart pill container and mobile phone APPs, we can also popularize the knowledge of (1) pharmacokinetics and pharmacodynamics, (2) principles for the use of medication, (3) smart nursing measures of commonly adverse drug reactions and events, and (4) medication guidance for home and outdoor among the elderly.

## 4. Smart Geriatric Nursing in Mental Health Based on User Profile

Smart geriatric nursing for mental health means considering the common psychological states, needs, and problems among the elderly regarding geriatric mental health standard to help the elderly to understand, identify, and deal with common mental problems and mental disorders correctly. Consequently, family members, doctors, and nurses can find emotional sustenance methods to contribute a high quality of the elderly's life. Smart mental health care for the elderly based on the user profile system technology uses a geriatric user profile system technology as is shown in Figure 4. The user profile system is designed to digitize and automate information which consists of a model of the basic information, preference information, and dynamic change information of the elderly, by which we can get the geriatric user profile. After modelling the geriatric user profile, we can apply smart mental health care for the elderly. The smart geriatric nursing in mental health based on the user profile is shown in Figure 5.

### 4.1. User Profile System of the Elderly for Smart Nursing in Mental Health

The basic framework of the user profile system for smart geriatric nursing in mental health is described in Figure 4. Through information fusion theory and technology such as Dempster–Shafer evidence theory for uncertain information modelling and processing [51–53], the static data and dynamic data of the elderly care object can be fused and processed. Subsequently, the user label and its weight information are obtained. Finally, the user profile for the elderly is obtained.

The basic information of the elderly including personality characteristics comes from the general information of the elderly. The preference information of the elderly includes hobbies, educational level, and occupational status before and/or after retirement. The dynamic information of the elderly includes changes in their family life, new knowledge from learning in daily life, and the dynamic situation from the surroundings and friends.

### 4.2. Implementation of Smart Geriatric Nursing in Mental Health

The implementation of smart geriatric nursing in mental health includes two aspects of nursing. On the one hand, the user profile of the elderly using information technology in Figure 4 supplies information that can reflect the psychological status and needs of the elderly. On the other hand, through online and/or offline counseling for the elderly, we can monitor the mental health state of the elderly changing along with the time. The basis of counseling is the well-recognized professional scales. The psychological counseling for the elderly is based on scales such as the Geriatric Depression Scale (GDS) [22, 23], Roy Coping and Adaptation Processing Scale (CAPS-15) [24, 25], and Eysenck Personality Questionnaire (EPQ) [26, 27].

As shown in Figure 5, after obtaining the psychological characteristic information of the elderly extracted by the user profile system in Figure 4, combining with the results of psychological counseling for the elderly, personalized mental comfort activities can be recommended intelligently. Recommended activities that can effectively promote the mental health of the elderly include cultural activities, tourism projects, recreational activities, and cognitive training projects.

With the help of smart nursing technology, psychological counseling, and interview activities based on the user profile system of the elderly, smart geriatric nursing in mental health can be implemented and provide more targeted psychological counseling, emotional relief, sadness comfort, daily care, and emotional catharsis for the elderly. Consequently, the risk level and occurrence of depression (emotional handicap), anxiety disorders (seasonal affective disorder) and other mental disorders, and psychological problems can be reduced. In this way, smart geriatric nursing can help the elderly cope with life in a healthy psychological state and always feel at ease.

## 5. Smart Geriatric Nursing for Daily Life Based on Big Data in Health

Smart geriatric nursing for daily life means helping the elderly to pursue high quality of life with reasonable arrangement of daily life and helpful assistance. Basing on (1) the user profile information of the elderly provided by Figure 4, (2) healthy big data from remote monitoring of the elderly shown in Figure 2, and (3) mental health big data shown in Figure 5, smart geriatric nursing for daily life can greatly meet the physical and psychological needs of the elderly. Consequently, we can achieve the goal of smart geriatric nursing for daily life based on big data in health.

The framework of smart geriatric nursing for daily life based on big data in health is shown in Figure 6. Smart geriatric nursing for daily life includes but is not limited to (1) recommendation of outdoor activities with smart tour for the elderly [54, 55]; (2) research and recommendation of university courses for the elderly or collective activities for the elderly [56]; (3) recommendation of physical status-based dietary habits, food taboos, and perceptions [57, 58]; (4) healthy menu recommendation [59, 60]; (5) data-based physical exercises recommendation [61, 62]; (6) rest and sleep wisdom reminder; (7) antifall reminder; and (8) cooking safe with smart kitchen [63]. Smart geriatric nursing for daily life should cover the diet and nutrition, environment and life, safety, and activities of the elderly in their daily life.

## 6. Limitation

There are some limitations in the current work. In general, the framework of smart geriatric nursing designed in this paper is mainly based on an ideal situation with enough resources in a developed society. Currently, as a developing country, in China, it is hard to fully implement the framework, especially in the rural area of China. But we do believe that the proposed framework is a good idea for smart geriatric nursing.

The big data and user profile of the elderly are the basis of smart geriatric nursing in mental health and for daily life. However, how to manage the privacy during using the big data is a challenge. In fact, protection of peoples' privacy in big data area is a worldwide social problem. Security should be addressed cautiously.

Advanced technologies can be helpful for smart geriatric nursing. However, too many technologies in smart geriatric nursing can be a double-edged sword. On the one hand, technology cannot replace the people to overcome the depression in older adults with chronic conditions. On the other hand, there are limitations in smart geriatric nursing like the economic effectiveness, accessibility, and practicality of some advanced technologies [44].

## 7. Conclusions

The Healthy China (2019-2030) program puts forward an implementation map for Healthy China strategy made by the Chinese government. Inspired by advanced technologies and the plan of elderly health promotion in the Healthy China program, this paper explores the framework of smart geriatric nursing and contributes a possible technical solution to the aging society. Smart geriatric nursing in physical health can realize a better medical care with smart devices using the technology of IoT. Smart geriatric nursing in mental health based on user profile offers helpful and smart services to the elderly regarding their mental health. In addition, the scales could effectively reflect some aspects of the mental health status for the elderly, which offers helpful information to the medical staff. Smart geriatric nursing for daily life is based on big data in health and serves all needs of the elderly in their everyday life.

The following research of this paper includes but is not limited to (1) more detailed optimization of relevant procedures, methods, and norms of intelligent elderly care, based on cloud computing platform; (2) integration, realization, and collection of related information of big data about geriatric daily nursing by artificial intelligence algorithm instead of the Internet of Things; and (3) continuation of the optimization of related technology and method.

## Figures and Tables

**Figure 1:** The framework of smart geriatric nursing.

**Figure 2:** Remote real-time monitoring for physical health of the elderly.

**Figure 3:** Smart nursing for medication safety using the smart pill container.

**Figure 4:** User profile system of the elderly (adopted and modified from [18]).

**Figure 5:** Smart geriatric nursing in mental health based on the user profile.

**Figure 6:** Smart geriatric nursing for daily life based on big data for health.

## Data Availability

The data used to support the findings of this study are included within the article.

## Additional Points

*Ethical Considerations*. Ethical issues (including plagiarism, informed consent, misconduct, data fabrication and/or falsification, double publication and/or submission, and redundancy) have been completely observed by the authors.
